The article "Bilateral Decompressive Hemicraniectomy for Diffuse Cerebral Edema and Medically Refractory Elevated Intracranial Pressure in Aneurysmal Subarachnoid Hemorrhage: A Case Series" was published in 2021. Journal: Cureus.

# Bilateral Decompressive Hemicraniectomy for Diffuse Cerebral Edema and Medically Refractory Elevated Intracranial Pressure in Aneurysmal Subarachnoid Hemorrhage: A Case Series

**DOI:** 10.7759/cureus.18057

**Published:** 2021-09-17

**Authors:** Nathan Quig, Darshan Shastri, Daniel Zeitouni, Edward Yap, Deanna Sasaki-Adams

**Affiliations:** 1 Department of Neurosurgery, University of North Carolina at Chapel Hill, Chapel Hill, USA; 2 Department of Neurosurgery, University of North Carolina at Chapel Hill School of Medicine, Chapel Hill, USA

**Keywords:** decompressive hemicraniectomy, cerebral edema, elevated intracranial pressure, anuerysm, aneurysmal subarachnoid hemorrhage

## Abstract

Decompressive hemicraniectomy (DCHC) may be indicated in the setting of subarachnoid hemorrhage (SAH) complicated by persistent elevated intracranial pressure (ICP) that is refractory to medical interventions. Outcomes can be variable as indications for surgery can include focal hematomas, infarctions, and regional or diffuse edema.

Bilateral DCHC for medically refractory elevated ICP in the setting of SAH is not well described in the literature, and the viability of this option in terms of patient outcomes is unclear. We describe the cases of four patients with medically refractory ICP secondary to diffuse cerebral edema who underwent bilateral DCHC in the setting of SAH.

This is a retrospective case review of four patients with aneurysmal SAH who underwent bilateral DCHC for management of diffuse global edema resulting in medically refractory ICP.

We describe two patients who made impressive recoveries after bilateral DCHC and two patients who required significant continued care needs despite ICP control in all patients.

Bilateral DCHC is a viable option for control of refractory elevated ICP in SAH patients who develop diffuse cerebral edema. Bilateral DCHC in this setting can be considered after exhaustion of other therapeutic options.

## Introduction

The standard of care after the occurrence of an aneurysmal subarachnoid hemorrhage (SAH) is early treatment of the ruptured aneurysm with either surgical clip ligation or endovascular treatment followed by management of the clinical sequala of SAH. The post-operative or post-embolization clinical course of SAH can vary widely in severity, with equally variable outcomes [1,2]. Outcomes are heavily dictated by the presence and severity of secondary effects of SAH, including hydrocephalus, vasospasm, cerebral salt wasting, and elevated intracranial pressure (ICP), as well as other morbidities experienced by intensive care level patients. Patients who develop elevated ICP benefit from first-line treatment modalities such as cerebrospinal fluid (CSF) diversion via external ventricular drain (EVD) placement, sedation, pain management, and hyperosmolar therapy [2]. Patients with elevated ICP refractory to first-line treatments present a challenging clinical situation. Consideration in this setting may include a period of electroencephalogram (EEG) burst suppression or decompressive hemicraniectomy (DCHC). Burst suppression comes at the expense of losing the clinical neurological examination and detection of clinically significant vasospasm.

The article "Bilateral Decompressive Hemicraniectomy for Diffuse Cerebral Edema and Medically Refractory Elevated Intracranial Pressure in Aneurysmal Subarachnoid Hemorrhage: A Case Series" was published in 2021. Journal: Cureus.

DCHC is a well-studied surgical procedure as a means to reduce elevated ICP in the setting of ischemic stroke, intraparenchymal hemorrhage, and severe traumatic brain injury [3-5]. In SAH complicated by elevated ICP, previous literature describes a variable role of DCHC as indications can include pathologic sequala of SAH including focal hematomas, regional or global edema, and swelling from infarction [6-11]. These case series are variable in whether DCHC was performed primarily (during surgical clipping of an aneurysm) or secondarily (after the development of elevated ICP). Additionally, these case series report mostly unilateral DCHC for unilateral pathology, making robust conclusions regarding indications and outcomes for DCHC after SAH difficult.

To our knowledge, bilateral DCHC after SAH for global cerebral edema is not well described in the literature or is conflated within case series of DCHC mostly reporting unilateral DCHC for the management of a focal lesion. In this case series, we will outline the cases of four patients with medically refractory elevated ICP secondary to diffuse cerebral edema after SAH who underwent bilateral DCHC.

## Case presentation

Patient 1 was a 64-year-old female who presented as an HH4F4 (Hunt-Hess 4 and Fisher grade 4) SAH (Figure 1A). Given a poor examination on presentation, an EVD was placed. Subsequent angiogram revealed a large right pericallosal aneurysm that was judged not to be amenable to coil embolization (Figure 1B). She was taken emergently to the operating room (OR) for a bifrontal craniotomy and clip ligation. Post-operatively, she developed intermittently elevated ICP, which was managed with first-line interventions until her EVD developed a poor wave form with unreliable ICP measurements. A head CT demonstrated collapsed ventricles and diffuse edema. A Licox® ICP monitor (Integra, Billerica, Massachusetts, United States) was placed, which confirmed elevated ICP (>30mmHg), and a pentobarbital infusion was started. The patient’s ICP became resistant to pentobarbital infusion, and a decision was made to take the patient to the OR for removal of the bifrontal craniotomy and extension of the previous craniotomy into an extended bifrontal craniectomy (Figure 1C). Post-operatively, her ICP remained well controlled, with all measurements of less than 20mmHg. After a prolonged ICU admission, the patient’s neurological examination slowly improved, and she was ultimately discharged to a skilled nursing facility after placement of a tracheostomy and gastrostomy tube (G-tube). At the six-month follow-up, the patient’s tracheostomy and G-tube had been removed, but she remained with a modified Rankin score (mRS) of 4.

The article "Bilateral Decompressive Hemicraniectomy for Diffuse Cerebral Edema and Medically Refractory Elevated Intracranial Pressure in Aneurysmal Subarachnoid Hemorrhage: A Case Series" was published in 2021. Journal: Cureus.

**Figure 1:** Imaging related to the clinical course of patient 1. (A) Head CT obtained on presentation demonstrated SAH secondary to a ruptured right pericallosal aneurysm. (B) Angiogram obtained after presentation demonstrating a large right pericallosal aneurysm. (C) Post-operative head CT after bilateral DCHC for refractory elevated ICP. SAH, subarachnoid hemorrhage; DCHC, decompressive hemicraniectomy; ICP, intracranial pressure

Patient 2 is a 48-year-old female who presented as an HH3F3 SAH secondary to a basilar tip aneurysm (Figure 2A). On arrival, an EVD was placed and the basilar tip aneurysm was successfully embolized with coils (Figure 2B). Initially, the patient had intermittent elevated ICP that was effectively managed with first-line interventions. On post-embolization day 6, the patient developed sustained refractory elevated ICP (>30mmHg), and a head CT demonstrated diffuse cerebral edema. A pentobarbital infusion was started, to which ICP remained refractory elevated. She was then taken to the OR for a bilateral DCHC (Figure 2C). Her ICP remained well controlled post-operatively. After a prolonged ICU stay complicated by vasospasm, she was discharged to a rehabilitation facility. At the nine-month follow-up, she was living at home independently with an mRS of 1 and requested clearance to return to work.

**Figure 2:** Imaging related to the clinical course of patient 2. (A) Head CT obtained on presentation demonstrated SAH secondary to a ruptured basilar tip aneurysm. (B) Angiogram obtained after presentation demonstrating a basilar tip aneurysm. (C) Post-operative head CT after bilateral DCHC for refractory elevated ICP. SAH, subarachnoid hemorrhage; DCHC, decompressive hemicraniectomy; ICP, intracranial pressure

Patient 3 is a 34-year-old female who presented as an HH3F4 SAH secondary to an anterior communicating aneurysm rupture (Figure 3A). On arrival, an EVD was placed and the aneurysm was successfully coiled (Figure 3B). On post-embolization day 10, she developed elevated ICP that was resistant to first-line intervention, and a head CT revealed diffuse cerebral edema. ICP remained refractory to a subsequent pentobarbital coma, and the patient was then taken to the OR for a bilateral DCHC. ICP remained well controlled post-operatively. After a prolonged ICU and hospital admission, her tracheostomy and G-tube were removed, and she was discharged to a rehabilitation facility with an mRS of 2. Unfortunately, she died five months later from complications of a urinary tract infection.

The article "Bilateral Decompressive Hemicraniectomy for Diffuse Cerebral Edema and Medically Refractory Elevated Intracranial Pressure in Aneurysmal Subarachnoid Hemorrhage: A Case Series" was published in 2021. Journal: Cureus.

**Figure 3:** Imaging related to the clinical course of patient 3. (A) Head CT obtained on presentation demonstrated SAH secondary to a ruptured anterior communicating artery aneurysm. (B) Angiogram obtained after presentation demonstrating an anterior communicating artery aneurysm. (C) Post-operative head CT after bilateral DCHC for refractory elevated ICP. SAH, subarachnoid hemorrhage; DCHC, decompressive hemicraniectomy; ICP, intracranial pressure

Patient 4 is a 55-year old female that presented as an HH4F3 SAH secondary to a presumed anterior communicating aneurysm rupture (Figure 4A). On arrival, an EVD was placed and an angiogram demonstrated a large irregular anterior communicating artery aneurysm as well as a left middle cerebral artery aneurysm (Figure 4B). She was then taken to the OR for an orbitozygomatic craniotomy for clip ligation of the two aneurysms. On post-operative days 1-5, she had elevated ICP that was responsive to first-line therapy. On post-operative day 6, a pentobarbital infusion was started for refractory ICP, which was unsuccessful. She was taken to the OR for a bifrontal and left DCHC (Figure 4C). After the DCHC, the patient’s ICP was remained controlled. After a prolonged course, she was discharged to a skilled nursing facility with an mRS of 4. She is now followed up annually to monitor an MCA aneurysm but is doing well at the skilled nursing facility. At her last follow-up (20 months post-aneurysm rupture), she was fully oriented and able to easily follow commands.

**Figure 4:** Imaging related to the clinical course of patient 4. (A) Head CT obtained on presentation demonstrated SAH secondary to a presumed anterior communicating artery aneurysm. (B) Angiogram obtained after presentation demonstrating an anterior communicating artery aneurysm and left middle cerebral artery aneurysm. (C) Post-operative head CT after bilateral DCHC for refractory elevated ICP. SAH, subarachnoid hemorrhage; DCHC, decompressive hemicraniectomy; ICP, intracranial pressure

## Discussion

SAH is a devastating disease, with an approximately 30% mortality rate within the first 28 days after ictus. Half of surviving patients can be left with permanent disabilities as a result of secondary injury resulting from the SAH [6]. If the secondary sequelae are identified early and managed aggressively, outcomes may be improved for patients. Elevated ICP is a relatively common clinical feature of high-grade SAH, which often responds to first-line therapies such as CSF diversion, sedation, and hypertonic saline. However, a small subset of patients can experience refractory elevated ICP requiring interventions beyond first-line treatments, such as a burst suppression with a pentobarbital coma. However, a pentobarbital coma comes at the expense of detecting clinical significant vasospasm, which has an actionable and potentially reversible course with aggressive treatment. Additionally, the risk/benefit decision of subjecting a critically ill patient to the well-known detrimental systemic side effects of pentobarbital can be a difficult decision to make.

The article "Bilateral Decompressive Hemicraniectomy for Diffuse Cerebral Edema and Medically Refractory Elevated Intracranial Pressure in Aneurysmal Subarachnoid Hemorrhage: A Case Series" was published in 2021. Journal: Cureus.

In this report, we described the cases of four patients where bilateral DCHC was utilized as a subsequent means of controlling refractory elevated ICP in the setting of diffuse cerebral edema following SAH. DCHC in the setting of SAH is described in the literature infrequently and often in the setting of unilateral pathology. Güresir et al. evaluated 860 patients with aneurysmal SAH and found a favorable outcome in 21 (26.6%) of the 79 patients who underwent DCHC, concluding that the timing of decompression was crucial to favorable outcomes [8]. Otani et al. studied 110 consecutive poor-grade SAH patients and found that in patients with unilateral space-occupying hematomas, urgent decompression led to favorable outcomes [6]. In a series of 964 patients with SAH undergoing decompression by Dorfer et al., underlying pathology significantly influenced outcomes with patients with increased intracranial hypertension from ischemic infarcts not receiving the same benefit from decompression as patients with hematoma-related brain swelling [7]. Goedemans et al. found that DCHC was associated with high rates of unfavorable outcomes overall but better outcome profiles in the setting of hematoma or edema as opposed to infarction [9]. Schirmer et al. reported reduced mortality when the decompression was performed on the non-dominant side and early [10]. D'Ambrosio et al. demonstrated benefits to short-term survival if DCHC was performed early but poor outcomes overall in this setting [11].

In our case series of four patients, maximal medical management was judged to have been achieved before the decision to pursue bilateral DCHC. Additionally, in each situation, unilateral DCHC was felt to be an inadequate option given the diffuse nature of the cerebral edema demonstrated on pre-operative head CT. Little data regarding the efficacy of this situation are available, making a detailed and informed conversation with the patient’s medical decision-maker(s) necessary. Of note, the patients in our series also underwent bilateral DCHC after initiation and failure of pentobarbital coma. In this setting, the role of proceeding with bilateral DCHC prior to initiation of pentobarbital is unclear but may be of benefit if the diffuse nature of edema and resultant elevated ICP is not expected to be adequately addressed with burst suppression.

The article "Bilateral Decompressive Hemicraniectomy for Diffuse Cerebral Edema and Medically Refractory Elevated Intracranial Pressure in Aneurysmal Subarachnoid Hemorrhage: A Case Series" was published in 2021. Journal: Cureus.

Though our case series is certainly limited in number, large-scale case series or trials are likely not feasible given the relative infrequent nature of this clinical situation. However, our case series suggest that bilateral DCHC in the setting of global diffuse cerebral edema following SAH is feasible with good outcomes possible. Two of the patients made quite impressive recoveries with discharge to acute inpatient rehabilitation facility and eventually home. On a follow-up clinic appointment, they had an mRS of 1 and 2. Two of the patients were discharged to skilled nursing facilities with an mRS of 4.

## Conclusions

In this case series, we reported four SAH patients with medically refractory ICPs secondary to global cerebral edema who underwent bilateral DCHC. Two of the four patients demonstrated impressive recoveries ultimately returning home after rehabilitation with mRSs of 1 and 2. The other two patients demonstrated poorer outcomes, even after successful control of ICP after bilateral DCHC. As such, bilateral DCHC may be a viable option for ICP control after the exhaustion of other therapeutic options in this setting. Patient selection is likely paramount and should be reserved for those who have exhausted other options and demonstrate global pathology. While our case series is small, larger case series or trials may be unlikely to materialize in the literature given the rarity of this clinical situation.
